The article "Role of NADPH Oxidase and Xanthine Oxidase in Mediating Inducible VT/VF and Triggered Activity in a Canine Model of Myocardial Ischemia" was published in 2014. Journal: Int J Mol Sci.

# Role of NADPH Oxidase and Xanthine Oxidase in Mediating Inducible VT/VF and Triggered Activity in a Canine Model of Myocardial Ischemia

**DOI:** 10.3390/ijms151120079

**Published:** 2014-11-04

**Authors:** James B. Martins, Ashok K. Chaudhary, Shuxia Jiang, Michael Kwofie, Prescott Mackie, Francis J. Miller

**Affiliations:** Division of Cardiovascular Diseases, Departments of Internal Medicine, University of Iowa and Veterans Affairs Medical Center, Iowa City, Iowa 52242, IA, USA; E-Mails: ashok-chaudhary@uiowa.edu (A.K.C.); shuxia-jiang@uiowa.edu (S.J.); michael-kwofie@uiowa.edu (M.K.); prescott-mackie@uiowa.edu (P.M.); francis-miller@uiowa.edu (F.J.M.)

**Keywords:** ventriculartachycardia/fibrillation, triggered activity, myocardial ischemia, NADPH oxidase

## Abstract

Background: Ventricular tachycardia or fibrillation (VT/VF) of focal origin due to triggered activity (TA) from delayed afterdepolarizations (DADs) is reproducibly inducible after anterior coronary artery occlusion. Both VT/VF and TA can be blocked by reducing reactive oxygen species (ROS). We tested the hypothesis that inhibition of NADPH oxidase and xanthine oxidase would block VT/VF. Methods: 69 dogs received apocynin (APO), 4 mg/kg intraveneously (IV), oxypurinol (OXY), 4 mg/kg IV, or both APO and OXY (BOTH) agents, or saline 3 h after coronary occlusion. Endocardium from ischemic sites (3-D mapping) was sampled for Rac1 **(**GTP-binding protein in membrane NADPH oxidase) activation or standard microelectrode techniques. Results (mean ± SE, * *p* < 0.05): VT/VF originating from ischemic zones was blocked by APO in 6/10 *, OXY in 4/9 *, BOTH in 5/8 * or saline in 1/27; 11/16 VT/VFs blocked were focal. In isolated myocardium, TA was blocked by APO (10^−6^ M) or OXY (10^−8^ M). Rac1 levels in ischemic endocardium were decreased by APO or OXY. Conclusion: APO and OXY suppressed focal VT/VF due to DADs, but the combination of the drugs was not more effective than either alone. Both drugs inhibited ischemic Rac1 with inhibition by OXY suggesting ROS-induced ROS. The inability to totally prevent VT/VF suggests that other mechanisms also contribute to ischemic VT.

## 1. Introduction

Ventricular tachycardia/ventricular fibrillation (VT/VF) due to myocardial ischemia is a major cause of cardiac arrest, a public health problem. Present therapies for preventing ischemic VT/VF are unsatisfactory and unsafe. Understanding the mechanisms underlying ischemic VT/VF is necessary to develop new and improved therapies. We have developed a clinically relevant canine model of ischemic VT/VF, which is mapped in 3-D and reproducibly stable in the same animal, thereby allowing for the testing of drug interventions and for collection of tissue from endocardial foci for subsequent study by standard micro-electrodes. We have shown that oscillations in cell membrane potential termed delayed afterdepolarizations (DADs), which give rise to endocardial or Purkinje triggered activity (TA) are found more commonly at the endocardial focus of VT [1]. Furthermore, drugs such as lovastatin [2], whose pleiotropic effects include reduction of reactive oxygen species (ROS), prevent DADs and TA *in vitro* and focal VT/VF *in vivo*. Regions of ischemic myocardium associated with focal VT can exhibit increased levels of ROS and scavenging of ROS prevented TA [3]. There are multiple potential enzyme systems responsible for generation of myocardial ROS. In this study, we tested the hypothesis that selective and potent inhibition of NADPH oxidase or of xanthine oxidase, two distinct enzymes capable of ROS production, would inhibit ischemic VT/VF. Despite blockade of TA at micromolar concentrations, we did not see greater anti-arrhythmic effects of these drugs even when administered simultaneously.

The article "Role of NADPH Oxidase and Xanthine Oxidase in Mediating Inducible VT/VF and Triggered Activity in a Canine Model of Myocardial Ischemia" was published in 2014. Journal: Int J Mol Sci.

## 2. Results

### 2.1. Summary Data

Of the 54 dogs studied after coronary occlusion, ten were randomly treated with apocynin (APO), nine with oxypurinol (OXY), eight with APO and OXY simultaneously (BOTH) and 27 concomitantly studied with saline. The latter served as ischemic controls for VT/VF inducibility over the time after coronary artery occlusion. Table 1 shows summary data for all treated VT/VF demonstrating comparable data except for inducibility. Dogs without drug treatment continued to have inducibility except for one (C23) throughout the test period while drug treatment resulted in non-inducibility in 15 of which 11 had focal mechanisms and 7 had reentry. The focal mechanisms were 83% endocardial and 17% epicardial while reentry was endocardial in 29% and epicardial in 71%. All mechanisms of VT/VF originated from ischemic or border zones. VF occurred equally before and after interventions including saline. VT/VFs with multiple mechanisms accounted for half or less of responses to drug. Non-sustained episodes, usually the result of drug intervention (Table 2, Table 3 and Table 4) lasted an average of 4 s.

### 2.2. Data for Apocynin (APO)

In the APO-treated group (Table 1 and Table 2), six dogs with focal VT/VF had induction blocked. Two of the latter had coexisting reentry blocked as well, but no experiment with only a reentry mechanism showed block. The dogs with reentry block (A4 and A9) also had VF. The response to APO was significantly different than dogs with ischemia and saline treatment with block of focal mechanisms accounting for the anti-arrhythmic effect of APO.

The article "Role of NADPH Oxidase and Xanthine Oxidase in Mediating Inducible VT/VF and Triggered Activity in a Canine Model of Myocardial Ischemia" was published in 2014. Journal: Int J Mol Sci.

**Table 1:** All group data.

DATA		APO	C	OXY	C	BOTH	C
**N (VT/VF)**		10	10	9	9	8	8
**Focal**		6 *	0	2 *	0	3 *	0
**Reentry**		2 ^†^	0	3 ^†,^*	0	2	1
**Total**		6/10 *	0/10	4/9 *	0/9	5/8 *	1/8
**AP**	sys	130 ± 5	132 ± 9	119 ± 9	116 ± 11	122 ± 9	114 ± 9
	dias	85 ± 8	83 ± 8	75 ± 8	74 ± 4	78 ± 6	76 ± 6
**ERP**		157 ± 4	156 ± 3	154 ± 6	154 ± 7	146 ± 7	148 ± 6
**Inf. size**		42 ± 8	48 ± 5	49 ± 7	47 ± 7	42 ± 12	42 ± 8

Abbreviations: APO, apocynin (4 mg/kg intravenneous (IV) after ischemia); C, ischemia control; OXY, oxypurinol (4 mg/kg IV after ischemia); BOTH, apocynin and oxypurinol given after ischemia; N, number experiments with VT/VF; Focal, number with that mechanism blocked; Reentry, number blocked; * *p* < 0.05 *vs.* ischemic controls; **^†^**, includes dogs with focal and reentrant mechanisms in one episode, see Table 2, Table 3 and Table 4; AP, arterial pressure; sys, systolic; dias, diastolic; ERP, effective refractory period (average of normal zones paced); Inf. size, Infarct size (% of risk zone), ±SE.

### 2.3. Data for Oxypurinol (OXY)

With OXY treatment (Table 1 and Table 3) two of four dogs had focal VT/VF blocked. In contrast to the APO group, dogs O1, O4 and O9 had endocardial reentry blocked. In OXY experiments, block of endocardial focal and reentry mechanisms was observed.

### 2.4. Data for BOTH (APO and OXY)

Treatment with BOTH agents (Table 1 and Table 4) blocked 3 of 4 focal mechanisms, including B1 the experiment highlighted in Figure 1 and Figure 2. In other dogs, only two of four endocardial reentrant abnormal QRS tachycardias (VTs) were blocked. Thus BOTH agents blocked focal mechanisms only, but not more effectively than either agent alone.

**Table 2:** Apocynin (APO) group details.

Dog #	SI	Mech	SII	Mech	AIII	Mech	AIV	Mech	Dog #	SI	Mech	SII	Mech	SIII	Mech	SIV	Mech
A1	VT	**EpFo**	VT	**EpFo**	NI	–	NI	–	C1	VT	EpFo	VT	EpFo	VT	EFo	VT	EpFo
A2	VF	EFo/RE	VF	EFo/RE	VF	EFo/R	nd	–	C2	VF	R	VT	R	VT	R	nd	–
A3	VF	**EFo/**RE	VT	**EFo**	NI	–	nd	–	C3	VT	R	VT	R	VT	R	VT	R
A4	VT	**EFo/R**	VT	**EFo/R**	VT ns	EFo	NI	–	C4	VT	R	VT	R	VT	R	VT	R
A5	VT	EFo	VT	EFo	VT	EFo	VF	EFo/RE	C5	VT	R	VT	R	VT	R	VT	R
A6	VF	EFo/RE	VF	EFo/R	VF	EFo	VT	EFo/R	C6	VF	EFo/R	VT	EFo	VF	EpFo	VT	EFo
A7	VF	EpFo/R	VF	EpFo/R	VF	EFo/R	VT	EpFo/R	C7	VF	EFo/R	VF	EFo/R	VF	EFo/R	VF	EFo/R
A8	VT	**EFo**	VF	**EFo**/R	VT ns	**EFo**	VT ns	**EFo**	C8	VF	EFo/R	VF	EFo/RE	VT	EpFo/RE	VT	EFo/R
A9	VT	**EFo**/**R**	VF	**EFo/R**	NI	–	VT ns	**EFo**	C9	VT	R	VT	RE	VF	EFoRE	VT	R
A10	VF	**EFo**	VF	**EFo/**RE	VT	**EFo**	NI	**–**	C10	VF	EFo	VF	EFo/RE	VF	EFo/RE	VF	EFo/R

Dog # given saline (S) for inductions I–II and Apocynin (A) or S for III and IV; ventricular tachycardia (VT); ventricular fibrillation (VF); Mechanism of sustained VT/F (Mech); endocardial focal (EFo); epicardial focal (EpFo); epicardial reentry (R); endocardial reentry (RE); Not inducible (NI); not done (nd); non-sustained (ns); C, ischemia control; and mechanism becoming non-inducible (shown in BOLD).

The article "Role of NADPH Oxidase and Xanthine Oxidase in Mediating Inducible VT/VF and Triggered Activity in a Canine Model of Myocardial Ischemia" was published in 2014. Journal: Int J Mol Sci.

**Table 3:** Oxypurinol (OXY) group data.

Dog #	SI	Mech	SII	Mech	OIII	Mech	O IV	Mech	Dog #	SI	Mech	SII	Mech	SIII	Mech	SIV	Mech
O1	VF	EFo**/RE**	VF	EFo**/RE**	VT	EFo	VT	EFo	C11	VF	EFo/RE	VF	R	VF	EFo/RE	VF	EFo/RE
O2	VT	R	VF	RE	VT	RE	nd	–	C12	VT	R	VF	EpFo/R	VF	R	VF	R
O3	VT	R	VT	R	VT	R	VT	R	C13	VF	EpFo**/**R	VF	RE	VF	RE	VF	RE
O4	VT	**EFo/RE**	VT	**EFo/RE**	NI	–	NI	–	C14	VT	RE	VT	RE	VT	RE	VT	RE
O5	VF	RE	VF	R	VT	R	VF	R	C15	VF	EFo/R	VF	R	VF	R	VF	EFo/R
O6	VF	EFo	VT	EFo	VF	EFo	VF	EFo	C16	VF	R	VF	EFo/R	VF	EFo/RE	VF	R
O7	VF	R	VF	R	VT	RE	VT	EFo/RE	C17	VF	RE	VT	R	VF	R	VT	R
O8	VT	**EFo**	VF	**EFo/**RE	VF	R	VTns	R	C18	VT	EFo	VF	EFo/R	VT	EFo	VT	EFo
O9	VF	**R**	VF	**RE**	VF	**RE**	NI	–	C19	VF	EFo/RE	VT	R	VT	R	VT	R

Dog number (#) given saline (S) for inductions I–II and Oxypurinol (O) or S for III and IV; ventricular tachycardia (VT); ventricular fibrillation (VF); Mechanism of sustained VT/F(Mech) = endocardial focal (EFo); epicardial focal (EpFo); epicardial reentry (R); endocardial reentry (RE); Not inducible (NI); not done (nd); non-sustained (ns); C, ischemia control; and mechanism becoming non-inducible (shown in BOLD).

**Table 4:** BOTH (APO and OXY) group data.

Dog #	SI	Mech	SII	Mech	BIII	Mech	BIV	Mech	Dog #	SI	Mech	SII	Mech	SIII	Mech	SIV	Mech
B1	VT	**EpFo**/R	VT	**EpFo**/R	VT	R	VT	R	C20	VF	EFo/RE	VT	EFo/R	VT	EFo/R	VT	EFo/R
B2	VT	**EFo**	VT	**EFo**	VTns	**EFo**	NI	–	C21	VT	R	VT	R	VT	R	VT	R
B3	VT	R	VT	R	VT	R	nd	–	C22	VF	RE	VT	R	VT	R	VT	R
B4	VT	R	VT	R	VT	R	VT	R	C23	VT	**R**	VF	EFo/**R**	VF	EFo/**R**	VT	EFo
B5	VT	EFo	VT	EFo	VT	EFo	nd	–	C24	VT	EFo/R	VT	EFo/RE	VF	EFo/R	VT	EFo/R
B6	VT	**RE**	VT	**RE**	NI	–	NI	–	C25	VT	EpFo	VT	EpFo	VT	EpFo	VT	EpFo
B7	VT	**EFo**	VT	**EFo**	NI	–	NI	–	C26	VT	EFo/R	VT	EFo	VT	EFo	VT	EFo
B8	VF	EFo**/RE**	VF	**RE**	VF	EFo**/RE**	NI		C27	VF	EFo	VT	EFo	VT	EFo/R	VT	EpFo

Dog number (#) given saline (S) for inductions I–II and BOTH Apocynin and Oxypurinol (B) or (S) for inductions III–IV; Mechanism of sustained VT/F (Mech); endocardial focal (EFo); epicardial focal (EpFo); epicardial reentry (R); endocardial reentry (RE); Not inducible (NI); not done (nd); non-sustained (ns); C, ischemia control; and mechanism becoming non-inducible (shown in BOLD).

**Figure 1:** (**a**) Recordings from B1 (Table 4) showing two mechanisms of VT. From top to bottom are recordings from electrocardiogram (ECG) lead II for paced (*) complexes A (last drive stimulus) and B–E (4 extrastimuli) and 12 complexes of VT (F–Q) with endocardial (E-) midwall (M-) or epicardial (Ep-) electrograms from pacing site (-P) as well as west (-W), central (-C), north (-N), northeast (-NE), central east (-CE) and southeast (-SE), in the infarct zone producing this VT. Horizonal line (over E-SE) defines 200 ms. Intracardiac activations are marked with lower case letters a–q above each tracing. VT-F is produced by an endocardial focus and VT-H is due to endocardial reentry involving E-C and M-N (Figure 2). Note conduction block between E-C and M-N/E-N consistent with reentry. VT-L is due to reentry between E-CE and M-N despite surface ECG showing similar QRS. The epicardial focus (Ep-W) gives rise to VT-O (arrow). All sites of VT origin were ischemic. After BOTH drugs no focal VT/VF was induced, but reentry VT continued to be induced; (**b**) Electrograms from B1 (**a**) showing VT-H due to endocardial reentry (ER). Recordings are as 1a (larger labels same as **a**) with additional endocardial electrograms from extreme northwest (-NWW), extreme north (-NN), southwest (-SW), and south (-S) of the endocardial focal VT complex F (labeled A) and ER complex H (electrograms identified by arrows and activation sequences by lines). Note the conduction block between E-C and E-N which starts the reentry with circuitous activation around E-C and E-N (see Figure 2 complex H). The first stimulus (S) is complex E in 1a and the second is the next drive which does not capture; and (**c**) Electrograms from B1 (**a**) showing VT-O due to epicardial focal mechanism (EpFo). Epicardial recordings are as (**a**) and (**b**) showing VT complex O in (labeled A) with EpFo identified by arrows). Note all surrounding recordings (see Figure 2 complex O) activate by <50% of the cycle length. This VT was blocked by BOTH drugs.

The article "Role of NADPH Oxidase and Xanthine Oxidase in Mediating Inducible VT/VF and Triggered Activity in a Canine Model of Myocardial Ischemia" was published in 2014. Journal: Int J Mol Sci.

**Figure 2:** 3-D maps displaying endocardial (**lowest panel**) midwall (**middle panel**) and epicardial (**top panel**) site activation times (ms) before (-) and after onset of surface QRS for VT-F (**top left**), VT-H (**top right**). VT-L (**bottom left**) and VT-O **bottom right**). Numerical times can be compared with activation positions labeled “f, h, l and o” on Figure 1a–c. As shown in the vertical bar on the right of each layer, yellow indicates early sites (−25 to 15), red indicates intermediate sites and green indicates late sites. White indicates activation earlier than −25. “p” marks a Purkinje recorded site. Note the focal activation of VT-F on endocardium (–53) in white area, enclosed by blue rectangle. VT-H is reentrant on endocardium with −69 ms and subsequent activation thru that layer at −11, 39 and 60 ms, enclosed by the blue oval. VT-L shows reentry on endocardium at −38 with subsequent activation thru that layer at 21 and 105 ms, enclosed by blue oval. VT-O is epicardial focal (blue square in yellow area). This series of maps shows the complexity of induced VT/F in this ischemic model.

### 2.5. Data for Proarrhythmia

With regard to possible proarrhythmia, we administered APO (*n* = 3) OXY (*n* = 7) and BOTH (*n* = 5) to dogs which had at least four rounds of induction with extrastimuli with no VT/VF. One dog given OXY had reentry VT and one dog given BOTH had focal VT induced. Thus no clear evidence of proarrhythmia was observed over simple reproducibility.

### 2.6. In Vitro Data

In endocardium studied *in vitro*, TA occurred in both normal and ischemic tissues with the latter being more common [1]; TA was blocked (*n* = 17) by APO (10^−6^ M) with the average number reduced from 1.9 ± 2 to 0.1 ± 0.2 (*p* < 0.05). Action potential measures were unchanged including resting membrane potential (RMP) from −86 ± 5 to −84 ± 5 mV, action potential amplitude (APA) from 73 ± 3 to 66 ± 3 mV, action potential duration (APD) at 90% repolarization (APD90) from 234 ± 12 to 219 ± 14 ms, and APD at 50% repolarization from 165 ± 6 to 148 ± 10 ms after APO (10^−6^). Similarly OXY blocked average number of TA (*n* = 12) from baseline at 2.8 ± 2.6, to 2.3 ± 3.6 during OXY (10^−9^ M) to 0.9 ± 1.6 (*p* < 0.05) during OXY (10^−8^ M) to 0.6 ± 1 (*p* < 0.05) during OXY (10^−7^ M) to 0, and by OXY (10^−6^ M) to 0 (*p* < 0.05), and somewhat reversed by washing (TA at 0.3 ± 0.9) without altering ischemic action potentials (Table 5 and Figure 3). With ischemic tissue APD alternans is common as pacing cycle length is shortened. Its presence is unrelated to TA.

**Figure 3:** Four panels showing paced action potentials, with the last marked by arrows, induced delayed after-depolarization mediated triggered activity marked with triangles. **Top panel**: Baseline; **Second panel**: Superfused with oxypurinol 10^−9^ M; **Third panel**: Superfused with oxypurinol 10^−8^ M; and **Fourth panel**: After wash. Oxypurinol blocks TA at 10^−8^ M.

**Table 5:** *In vitro* action potential data for Oxypurinol.

DATA	Baseline	OXY 10^−9^	OXY 10^−8^	OXY 10^−7^	OXY 10^−6^	Wash
RMP (mV)	−77 ± 2	−75 ± 3	−77 ± 3	−77 ± 4	−69 ± 3	−79 ± 5
APA (mV)	73 ± 3	69 ± 3	71 ± 4	69 ± 4	63 ± 5	69 ± 10
APD90 (ms)	238 ± 14	238 ± 16	232 ± 16	231 ± 18	233 ± 20	215 ± 20
APD50 (ms)	169 ± 10	170 ± 12	163 ± 13	159 ± 15	166 ± 16	158 ± 18

Abbreviations: Resting membrane potential (RMP), action potential amplitude (APA), action potential duration (APD) at 90% repolarization (APD90), APD at 50% repolarization (APD50).

### 2.7. Rac1 Data

The activation of the small GTPase Rac1 is necessary for NADPH oxidase dependent generation of ROS [4]. Myocardial levels of active Rac1 were increased mildly although not significantly in ischemic endocardium (+) as compared to the nonischemic endocardium (−) from the same animals (Figure 4). In contrast, activated Rac1 in epicardium was not different. Treatment with APO or OXY dramatically reduced the levels of active Rac1 (Figure 4).

The article "Role of NADPH Oxidase and Xanthine Oxidase in Mediating Inducible VT/VF and Triggered Activity in a Canine Model of Myocardial Ischemia" was published in 2014. Journal: Int J Mol Sci.

**Figure 4:** (**A**) Western blots of active Rac1 and GAPDH (loading control) in endocardium (Endo) and epicardium (Epi) from animals after apocynin (APO) or oxypurinol (OXY) or no treatment with ischemia (control); Summary of active Rac1 levels in (**B**) endocardium and (**C**) epicardium from ischemic myocardium normalized to non-ischemic myocardium; and (**D**) the ratio of endocardial to epicardial Rac1 levels. Dogs pretreated with APO (*n* = 4) or OXY (*n* = 4) had reduced levels of active Rac1 compared to saline treated controls with ischemia (*n* = 12). * *p* < 0.05 *vs.* control.

## 3. Discussion

### 3.1. General

This investigation attempted to address the pathophysiology of acute ischemic VT/VF by attacking two separate pathways of cellular ROS production in myocardium. We had previously shown that ROS production contributed to arrhythmogenesis in our model since prior studies with less potent [3] or non-specific scavengers of ROS partially blocked VT due to TA [2]. In the present study we administered more potent drugs (blocking TA at 10^−8^ to 10^−6^ M), which individually blocked mainly focal VT/VF, but not more effectively than previously (LOVASTATIN at 10^−7^ M [2] or TEMPO at 10–10^−3^ M [3]). We expected both APO and OXY given simultaneously would prevent induced ischemic VT/VF to a greater extent, and that all focal, and perhaps reentry mechanisms, would be inhibited, but we found no greater effect.

### 3.2. In Vivo Model Considerations

Our model shows several mechanisms of ischemic VT/VF with the most common being endocardial focal as well as epicardial reentry, as also described by others in ischemic models [5]. Endocardial mechanisms are particularly interesting because of clinical results of ablation [6,7] prevent induction of VT and implantable defibrillator shocks. Even in acute infarction [8,9] VT can be successfully ablated with catheter-based techniques aimed at Purkinje or papillary muscles [10,11].

This model demonstrated complex mechanisms of *in vivo* VT/VF, which might be expected to resist anti-arrhythmic approaches. Indeed our data suggest that VF was especially associated with more than one underlying mechanism. Yet this complexity does not predict anti-arrhythmic failure, since prevention of one mechanism by inhibiting NADPH or xanthine oxidase, which occurred in 15 experiments, occurred by at least one episode with complex mechanisms in 12, resulting in non-inducibility in 9. Continued inducibility despite drug therapy (*n* = 12) simply reflects mechanisms which were not prevented regardless of complexity (only 5 of the 12). Clinically, prevention of a spontaneous VT/VF might also be due to an endocardial trigger which was eliminated by a treatment. Continued induction by extrastimuli occurring in an otherwise arrhythmia-free heart may mean that an induction protocol takes the place of an endocardial trigger.

The article "Role of NADPH Oxidase and Xanthine Oxidase in Mediating Inducible VT/VF and Triggered Activity in a Canine Model of Myocardial Ischemia" was published in 2014. Journal: Int J Mol Sci.

The most likely cause for failure of anti-arrhythmic agents in this series is that other non-ROS mediated mechanisms must play a role. An alternative explanation for failure to respond to drug intervention may include failure of the drug(s) to reach the ischemic focus. This is unlikely since the endocardial focus or reentry mechanisms probably involve tissues perfused by cavity blood or collateral blood flow. We had previously investigated this possibility showing that spontaneous VT in a 24 h old dog model showed similar slowing with intravenous as well as intra-coronary injections of metoprolol [12]. Also intravenous ZP123 blocked epicardial reentry in this same model [13] showing that drug can get to this risk zone site. Yet another alternative explanation for failure may be lack of appropriate concentration of the drug(s) to reach the ischemic focus, but our *in vitro* data showing efficacy of these drugs at 10^−6^ to 10^−8^ M make this unlikely. Therefore our data strongly support other non-ROS mediators in ischemic VT/VF.

### 3.3. In Vitro Correlations

Our *in vitro* data begs the question why all focal mechanisms would not be blocked. Several issues must be considered. First the *in vitro* TA was not sustained as was the *in vivo* VT/VF so the persistence at least raises the possibility of additional mechanisms, not only electrophysiological but also non-ROS mediated ones. So micro-reentry and mitochondrial mediated mechanisms, for example, may play a role. Additionally the superfusion with oxygenated Tyrode’s solution may produce a reperfusion-like state which may overemphasize the ROS mediated mechanisms. Nevertheless the *in vitro* data help to confirm the results *in vivo*, additionally excluding other electrophysiological effects of the drugs tested in a dose response fashion.

### 3.4. Effects of Defibrillation

We considered other possibilities of false VT/VF block with time by our concomitant groups of dogs with ischemia which had reproducible induction of the same arrhythmic mechanisms. In this series we observed the possibility of altered substrate only once in 27 experiments (C23) and therefore this is unlikely to explain the drug intervention data. Theoretically, the defibrillation of the second VF in C23 may have altered the arrhythmia substrate, owing to damage to myocardium by direct current shocks. Indeed experiments A8 and A9 may have appeared to respond to APO by becoming non-sustained after defibrillation. This explanation is unlikely because the group unresponsive to APO also had VF induced at least once in each of 5 as did 6 of the controls. Similar results occurred with OXY and BOTH. Thus VF and resultant defibrillation unlikely changed subsequent inducibility or mechanism.

The article "Role of NADPH Oxidase and Xanthine Oxidase in Mediating Inducible VT/VF and Triggered Activity in a Canine Model of Myocardial Ischemia" was published in 2014. Journal: Int J Mol Sci.

### 3.5. Mechanisms Involving Reducing Reactive Oxygen Species (ROS)

Mechanistic investigation of ischemic VT/VF has focused on ROS because of experimental observations [14,15,16,17,18,19,20,21]. Initial interest addressed heart function showing improvement [14,15,16,17] in ischemic models. Further studies showed antiarrhythmic effects [2,3,18,19] with variable results after apocynin [20] or oxypurinol [20,21]. Clinical trials have shown no benefit with antioxidants in multiple doses, but this failure may reflect a simple dose response problem and/or failure to inhibit ROS production. A more targeted approach of inhibiting the enzymes responsible for increased ROS has been proposed as a potential strategy and provides the rationale for this study.

Our data show that inhibiting NADPH oxidase (APO) or xanthine oxidase (OXY) was anti-arrhythmic in this model. It is possible that these two enzymes are activated independent of each other or in series. However, our data suggest the latter for several reasons. The first is that the inhibition of both pathways simultaneously did not totally prevent focal VT/VF. The second is the observation that whereas it was expected that APO inhibited activation of Rac1, we also observed that OXY partially inhibited Rac1 activation. This finding suggests that xanthine oxidase-derived ROS contributes to the activation of NADPH oxidase. The concept of ROS-induced ROS has been previously described in mediating arrhythmias in the intact heart [22], and implicate mitochondrial ROS. Multiple enzymatic sources of ROS, including NADPH oxidase and xanthine oxidase have been implicated in atrial fibrillation [21,23]. Finally other downstream mechanisms such Ca^2+^, Na^+^ or Na/Ca exchange channels [24,25,26,27] may also be responding to ryanodine receptor and/or calcium/calmodulin dependent protein kinase II activation [28]. Obviously more experiments are needed to address these hypotheses.

### 3.6. Limitations

Limitations of the model used for these studies involve an open-chest dog model with myocardial ischemia. Even with 23 plunge electrodes in the area of ischemic zone and surrounding recording up to 85 signals, we cannot exclude microreentry. Our data do show that drugs which block ROS production blocked focal VT/VF compared with reentry, but some tissues may not respond because of higher ROS or other mechanisms which are arrhythmogenic. Our studies support the latter possibility.

The article "Role of NADPH Oxidase and Xanthine Oxidase in Mediating Inducible VT/VF and Triggered Activity in a Canine Model of Myocardial Ischemia" was published in 2014. Journal: Int J Mol Sci.

We also recognize the limitations of the canine ischemic model because of variable and large collateral coronary circulation even visible to the naked eye. Clearly this may produce a more limited and endocardial ischemic zone, but this is, in fact, what is observed in humans who develop these collaterals over time of ischemic coronary disease, rendering human infarcts in that setting similarly smaller and endocardial [6,7,8,9,10,11]. Also we studied induced, not spontaneous VT/VF which may not have the same meaning as spontaneous VT/VF, however the anesthetized open chest state certainly adds additional confounding components. Finally the data reported herein focus on the immediate post occlusion state, which therefore only allows conclusions to apply to that specific time frame and not to others which may have additional mechanisms to assess.

## 4. Materials and Methods

### 4.1. Animals

Dogs weighing 12–20 kg of either sex were studied. The protocol was approved by the University of Iowa Animal Use and Care Committee and adhered to the standards of the American Physiological Society. Anesthesia was initiated with ketamine (5 mg/kg IM) and propofol (0.4 mg/kg intravenneous (IV)) and continued with α-chloralose given as a bolus (200 mg/kg). Constant infusion of α-chloralose (8 mg/kg/h,) was used to maintain anesthesia. The dogs were intubated and mechanically ventilated on a volume-cycled respirator (Harvard Apparatus, South Natick, MA, USA) to maintain a pO_2_ of 80–110 mmHg and a pCO_2_ of 35–45 mmHg. NaHCO_3_ was infused as necessary to maintain the pH range of (Radiometer, Copenhagen, Denmark). The femoral vein and artery were cannulated for administration of fluid and drugs and also for continuous measurement of mean arterial blood pressure. The sternum was sectioned in the midline to expose the heart for electrode placement to map VT/VF. The pericardium was incised and sutured to the wound edges forming support for the heart. A silk suture was passed under the left anterior descending coronary artery just distal to the first diagonal branch; the distance from the left atrial appendage was chosen greater than 10 mm to prevent inclusion of the first septal perforator in the risk zone. Epicardial temperature was maintained at ~37 °C by an infrared lamp and a plastic sheet draped over the sternotomy. Warm saline was applied to the heart intermittently to prevent surface drying.

The article "Role of NADPH Oxidase and Xanthine Oxidase in Mediating Inducible VT/VF and Triggered Activity in a Canine Model of Myocardial Ischemia" was published in 2014. Journal: Int J Mol Sci.

### 4.2. Electrophysiological Methods

Surface ECG leads (II and V5R) were recorded continuously. The right atrial appendage was stimulated at twice diastolic threshold with pulses of 2 ms duration with a bipolar electrode at > 200 b/min to control heart rates during all interventions. Ventricular cathodal pacing was performed on one pole of three multipolar transmural needles (see below) in non-risk zone sites with a 7 cm^2^ anode in the abdominal wall. We measured late LV diastolic threshold during each intervention by dialing the current down until failure to capture. However, for thresholds > 70 µA, other sites were chosen. Effective refractory period was measured by extra-stimuli [2,3].

### 4.3. Recording of Electrograms

Twenty-three plunge needle electrodes were placed into the anterior LV in and around the risk zone [2,3]. Electrodes were manufactured by J. Kassell (Fayetteville, NC, USA) with each pole completely surrounding the needle shaft to improve recording of adjacent muscle and Purkinje tissue. Bipolar electrograms were recorded sequentially down the needle via imaging from a synchronized storage oscilloscope during atrial pacing. The innermost bipolar pair was chosen with the earliest complex electrograms reflecting Purkinje (see below for definitions) and endocardial potentials from pairs immediately epicardial to the cavity potential. Midwall bipolar electrograms were recorded half way between the endocardium and epicardium. Epicardial electrograms were the latest activated on each multipole and nearly always recorded from the outer two electrodes. We utilized an array suited to the coronary anatomy; inter-needle distance varies over 6–10 mm.

### 4.4. Signal Detection, Ischemia Analysis and Mapping

Surface ECGs were recorded simultaneously with bipolar electrograms from up to 3 different sites on each of 23 16-pole electrodes by a personal computer based system with Matlab7.11 software interfaced with a high-speed data acquisition board (Microstar Laboratories, Bellevue, WA, USA) with its own 88000 processor, a 12-bit A/D converter and 96 kilobytes of SRAM [2,3]. The maximum sampling rate is 235 kHz. Each electrogram was amplified by a gain of 10–1000, band pass filtered between 3 and 1300 Hz, and sampled at 3200 Hz. Thus 64 independent instrument amplifiers are recorded for 14 s of data including 4 s before a selected manual trigger. The customized Matlab programs (MathWorks, Boston, MA, USA) control the acquisition, processing and visualization of the electrophysiological data.

The article "Role of NADPH Oxidase and Xanthine Oxidase in Mediating Inducible VT/VF and Triggered Activity in a Canine Model of Myocardial Ischemia" was published in 2014. Journal: Int J Mol Sci.

### 4.5. Ischemia Assessment

Ischemia analysis of individual tracings was categorized off line according to criteria selected first by algorithm and confirmed by the user. The algorithm selected maximum *dV*/*dt* within a window 30 ms before to 80 ms after the surface QRS onset as set by user. Then, an interval representing the actual local electrogram duration was calculated in steps. The interval margins were chosen as the points around the max *dV*/*dt*; (1) that proceeded forward to the isoelectric line and (2) backward to a specific factor of the average slope of the tracing. Within this local interval the maximum positive to maximum negative voltage was calculated. Ischemia was determined by at least a 45% drop in maximal total voltage from before to after coronary artery occlusion [29]. When the former criterion was borderline, ischemia by *dV*/*dt* was confirmed by an additional 45% decrease in this maximum slope.

### 4.6. Mapping

Mapping (activation) analysis was performed by a computer algorithm searching for max *dV*/*dt* applied off line and confirmed by hand. For each user chosen surface QRS, the algorithm scans all channels to distinguish “good” channels, which are used as templates for detecting signals for all other channels. A “good” channel is defined as an electrogram which has all signals spaced within 120 ms between onsets and intracardiac signals with peak amplitudes that are more than 60% of the average maximum of that channel. A “good” channel and its “good” neighbor will have max *dV*/*dt* detection within a 20 ms window of the peak amplitude found as above. Signals in all other “not good” electrograms are detected as max *dV*/*dt* within window spanning 40 ms before and 80 ms after for intracardiac onsets or 15 to 150 ms after pacing onset. All signal detection finds max *dV*/*dt* of smoothed electrogram (convolution MatLab function with averaging window = 50) then max *dV*/*dt* of original electrogram within +/− 8 ms of smoothed max. However, electrograms denoted as “good,” electrograms neighboring “good,” and all VF signals are detected with max *dV*/*dt* only (no smooth). Next, all intracardiac onsets are sequenced. An “adjacency” matrix is calculated for all electrodes. The adjacency matrix determines if calculated signals for each layer (endo, mid, epi) of an electrode are within a margin of each other. Starting at the first intracardiac onset, the margin encompasses +/−20 ms for neighboring layers (endo-mid, mid-epi) and +/−30 ms for endo-epi signals. Margins increase by 2 and 3 ms respectively for each following onset. The sequencing algorithm involves modifying the position of a signal that lies outside the margin of the signals of the two other layers. The outlier is moved by finding the max *dV*/*dt* within a window corresponding to a trend formed by the other signals. No sequencing is performed for VF onsets or pacing onsets. After all processing, each channel undergoes a refractory period check. All signals must occur at least 65 ms after the previous signal. If this is not satisfied, the signal will be recalculated in a time window of 80 ms starting 65 ms after previous signal. Isochrones are calculated and drawn by computer program.

The article "Role of NADPH Oxidase and Xanthine Oxidase in Mediating Inducible VT/VF and Triggered Activity in a Canine Model of Myocardial Ischemia" was published in 2014. Journal: Int J Mol Sci.

### 4.7. Definitions

Definitions [2,3] Reentrant VT: The electrode recording the earliest activity is located immediately adjacent to the site of the latest activation from the previous complex and continuous diastolic activity is frequently recorded between complexes (see Figure 1b). Electrograms are considered uninterpretable only if QRS to QRS reproducibility with pacing is not clear. There is no arbitrary exclusion based on voltage of electrograms, but short cycle lengths indicating refractory block are manifest by >75% reduction of voltage. Additionally, unidirectional block is associated with circuitous activation in adjacent sites and increased voltage of the subsequent activation on the electrogram showing block [5]. Refractory periods during tachycardia are assumed to be shorter in epicardium (80 ms) than endocardium (100 ms); these values are utilized by algorithm to consider reentry when present. Finally entrainment criteria suggesting reentry are present with overdrive pacing.

#### 4.7.1. Focal Ventricular Tachycardia (VT)

The electrode recording the site of origin is earliest and surrounded by other adjacent electrodes, which record progressive activation away from the origin, and no return to it as manifested by no late electrical activity (50% of the cycle length) on adjacent sites (see Figure 1c). This mechanism does not show entrainment.

#### 4.7.2. Purkinje Origin of Ventricular Tachycardia or Fibrillation (VT/VF)

A focal endocardial VT with recording of a Purkinje potential before the QRS on the endocardial electrogram recording the focus. To qualify, Purkinje electrograms must also be identified during atrial pacing by high frequency, low amplitude signals (0.5-mV spikes lasting 1–2 ms) recorded by multiple pairs of electrograms prior to endocardial muscle by 1–11 ms. The Purkinje potential also proceeds the atrial paced surface QRS recorded both before and after coronary artery occlusion.

#### 4.7.3. Sustained VT

A VT that does not stop on its own before 10 s or requiring pace termination or cardioversion/defibrillation to terminate. Non-sustained VT must last at least 3 complexes and less than 10 s to be considered an episode for mechanism.

The article "Role of NADPH Oxidase and Xanthine Oxidase in Mediating Inducible VT/VF and Triggered Activity in a Canine Model of Myocardial Ischemia" was published in 2014. Journal: Int J Mol Sci.

#### 4.7.4. VF

Tachycardia with changing surface QRS complex, which produces no arterial pressure requiring defibrillation to restore arterial pressure generation; analysis of the first 8–40 complexes allows reentry or focal mechanisms to be identified before multiple wavelets and out of array mechanisms take over.

### 4.8. Protocols

Experimental protocol and arrhythmia induction [2,3]: After confirming physiological blood gases, adequate anesthesia and quality electrogram recordings, the anterior descending artery was ligated permanently. Induction protocols are done 60 min later since infarct size in the open chest dog is then nearly maximal. We paced endocardium at apical septum and left ventricular base and lateral free wall just outside the risk zone to induce VT with up to four extrastimuli. After measuring the effective refractory period, the S_1_–S_2_ interval was prolonged by 5 ms and an S_3_ is added to the protocol initially with an S_2_–S_3_ interval equal to 50 ms >S_1_–S_2_. The intervals are shortened by 10 ms until either VT induction or failure to capture occurs. If VT is not induced, the S_2_–S_3_ interval is prolonged to capture and then third (S_4_) and fourth (S_5_) extrastimuli are added. When sustained VT occurs, attempts at pacing are performed to terminate the VT. Applying epicardial shocks of 20 J with a defibrillator also terminated VF. If no VT/VF is inducible after at least one hour of attempts (about every 15 min) then VT/VF will not likely be induced later [30]. The drugs listed below were then infused to address proarrhythmia potential.

When inducible VT/VF occurred, reproducibility was shown when two VTs with the same morphology or VFs were induced separated by 15 min [2,3]. Then drugs were infused over 10 min to attempt blockade of VT/VF induction. Drugs included were the NADPH oxidase inhibitor apocynin (APO, 4 mg/kg IV), the xanthine oxidase inhibitor oxypurinol (OXY, 4 mg/kg IV), BOTH (4 mg/kg IV each), or saline. Five min after the infusion, extra-stimulus testing was started from each site(s), which had previously produced reproducible VT. Block of sustained VT/VF was defined as failure to re-induce a reproducible mechanism with the same extra-stimulus protocol and one additional extra-stimulus; this result could occur immediately after administration of drug or after the second induction. Non-sustained VT, which terminates on its own in less than 10 s, was also considered non-inducibility. These non-inducible endpoints were demonstrated for a minimum of 30 min prior to concluding that the drug prevented VT/VF induction [2,3].

### 4.9. Intracellular Recording Techniques

After 3-D mapping, which identified either foci of Purkinje/endocardial VT origin or endocardial ischemic sites, endocardium was studied in an isolated tissue bath utilizing the following techniques [1,2,3]. The heart was excised and placed in ice-cold Tyrode’s solution with the selected electrode(s). The solution was equilibrated with 95% O_2_, 5% CO_2_ and contained (in mM) 125 NaCl, 24 NaHCO_3_, 2.7 KCl, 2.7 CaCl_2_, 0.5 MgCl_2_, and 0.25 Na_2_HPO_4_ and 5.5 dextrose (pH 7.4). Tissue measuring 4 × 3 × 2 mm^3^ (length × width × thickness) was removed from the area of the electrode beneath the surface of the solution. It was then placed in the bath, endocardium up, perfused with oxygenated Tyrode’s solution at 37 °C with a bath volume of 3 mL and perfused at a rate of 6 mL/min allowing the contents to be changed twice per minute. The tissue was stimulated with a bipolar electrode placed directly on it, pacing at 2 times diastolic threshold. Superficial fibers were impaled with 3 M KCl filled glass capillary microelectrodes with tip resistances measured from 3 to 20 MΩ. Microelectrodes were connected to a high input impedance preamplifier having capacity neutralization (AxoClamp, 2A Axon Instruments, Foster City, CA, USA) and the tissue bath grounded with a Ag-AgCl pellet.

The article "Role of NADPH Oxidase and Xanthine Oxidase in Mediating Inducible VT/VF and Triggered Activity in a Canine Model of Myocardial Ischemia" was published in 2014. Journal: Int J Mol Sci.

Action potentials (APs) were displayed on an oscilloscope and stored on a computer with pClamp (Molecular Devices, Sunnyvale, CA, USA,) software with data filtered at 1 kHz and sampled at 2 kHz. Maximum diastolic potential (MDP) in mV was measured as the average voltage just before the stimulus artifact of 10 paced complexes at a frequency of 1.5 Hz. Action potential amplitude (APA) in mV was measured as the average voltage from the MDP to the peak of the phase 1 of 10 paced complexes at a frequency of 1.5 Hz. Action potential durations (APD) at 50% and 90% repolarization from MDP were measured with the cursors of the clampan software of pClamp. Additional measurements were made using different pacing protocols with cycles (1–4 Hz) of an average of 30 s and abrupt cessation. Gradual phase 4 depolarization was recorded when continuing depolarization occurred over the course of 10 s whether or not spontaneous action potentials occurred. DADs (delayed after depolarizations) were defined as transient membrane decreases and repolarizations, occurring after full repolarization of the last paced AP. TA (triggered activity) was defined as a full AP occurring at the peak of a DAD. After reproducibility defined by TA that were stimulated on at least pacing drives, repeat stimulation was then performed with interventions including: (1) normal solution alone or with isoproterenol (5 × 10^−7^ M) to promote TAs; (2) drug intervention (apocynin, 10^−6^ M or oxypurinol 10^−9^ to 10^−6^ M) with repeat stimulation after 5 min superfusion and (3) after 20–30 min of washing with Tyrode’s and/or isoproterenol alone to determine reversibility. These tissues are remarkably stable showing only gradual improvement as superfusion continues for several hours [1,2,3]. Each dose of drug was evaluated by total numbers of TA produced with pacing of at least 4 frequencies divided by the number of trials.

The article "Role of NADPH Oxidase and Xanthine Oxidase in Mediating Inducible VT/VF and Triggered Activity in a Canine Model of Myocardial Ischemia" was published in 2014. Journal: Int J Mol Sci.

### 4.10. Measurement of Active Rac1

Following 3-D mapping, ischemic and nonischemic sites were collected and divided into epicardial and endocardial segments. Activation of the small GTPase Rac1 was measured by p21-activated protein kinase 1 pull-down assay according to the manufacturer’s recommendations (Enzo Life Sciences, Inc., Farmingdale, NY, USA). This assay uses a GST-fusion protein containing the p21-binding domain (PBD) of human p21-activated kinase 1 (Pak1) to affinity precipitate active Rac1 (GTP-Rac1) from the tissue lysates. The pulled-down active or GTP-Rac1 was detected by Western blot analysis using Rac1 antibody. Blots were imaged and densitometry quantitated with Odyssey SA Imaging System and Image Studio Software (Li-Cor Biosciences, Lincoln, NE, USA). GTP-Rac1 was normalized to GAPDH. Mean data from ischemic areas were normalized to mean data of the non-ischemic area.

### 4.11. Statistics

The effect of drug treatment on the incidence of VT/VF was evaluated by Chi Square. DADs and TA were analyzed by a two-tailed Fisher’s exact test at each dose level. The effect of these drugs on effective refractory period and arterial pressure was analyzed by a two-way ANOVA with repeated measurements. Rac1 data was analyzed by ANOVA with Tukey’s *post hoc* analysis. *p* < 0.05 was considered statistically significant. All values are reported as mean ± SE
